# LINC-DUBR Suppresses Malignant Progression of Ovarian Cancer by Downregulating miR-107 to Induce SMAC Expression

**DOI:** 10.1155/2022/4535655

**Published:** 2022-03-03

**Authors:** Zhehui Han, Dan Li, Yun Yang, Hong Zhang

**Affiliations:** ^1^Department of Gynecology, Tianjin Central Hospital of Gynecology and Obstetrics, Tianjin Key Laboratory of Human Development and Reproductive Regulation, Maternity Hospital of Nankai University, Tianjin 300000, China; ^2^Department of Gynecologic Oncology, Tianjin Central Hospital of Gynecology and Obstetrics, Tianjin Key Laboratory of Human Development and Reproductive Regulation, Maternity Hospital of Nankai University, Tianjin 300000, China

## Abstract

**Background:**

LINC-DUBR may be a potential therapeutic target in ovarian cancer (OC). The purpose of this research was to explore the impact of miR-107 on the tumorigenicity of OC and its underlying molecular mechanisms.

**Methods:**

RT-qPCR was adopted to measure the expression of LINC-DUBR and miR-107 in ovarian cancer tissues and cells. CCK-8 assays and transwell chamber assays were conducted to evaluate the impacts of LINC-DUBR and miR-107 on the proliferation and invasion of human ovarian cancer cells (SKOV3). In addition, we determined the relationship between LINC-DUBR, miR-107, and SMAC using TargetScan and luciferase reporter assay. The protein expression of SMAC was determined by western blot.

**Results:**

Compared with normal tissues and cells, LINC-DUBR was downregulated and miR-107 was highly expressed in ovarian cancer tissues and cell lines. Overexpression of LINC-DUBR inhibited the cell proliferation and invasive ability in OC cells SKOV3. The luciferase reporter assay proved overexpression of LINC-DUBR repressed cells proliferation and invasion via binding to miR-107 in ovarian cancer. In addition, we found that SMAC was downregulated directly by miR-107 in ovarian cancer. miR-107 mimic significantly increased cell proliferation and invasiveness of SKOV3, while overexpressed SMAC eliminated this effect. Furthermore, miR-107 could regulate the XIAP/caspase-3 signaling pathway in ovarian cancer by targeting SMAC.

**Conclusion:**

LINC-DUBR suppressed malignant progression of ovarian cancer by downregulating miR-107 to induce SMAC expression and involving in the XIAP/caspase-3 signaling pathway.

## 1. Introduction

Ovarian cancer (OC) accounts for a high proportion of female reproductive system related diseases, which seriously affects women's health. Ovarian cancer has a high incidence and poor prognosis for patient survival. In 2018, there were 52,100 new ovarian cancer patients and 22,500 dead patients in China [1]. Ovarian cancer is not easy to be found in the early stage. When patients go to the hospital for diagnosis, most of them are in the advanced stage. At present, surgery combined with radiotherapy and chemotherapy is the most common measure to treat ovarian cancer, but the treatment effect is not satisfactory. It is essential to deeply explore the pathogenesis and determine new therapeutic targets of ovarian cancer.

lncRNA is a noncoding RNA consisting of over 200 nucleotides and cannot encode protein [2, 3]. It widely exists in the transcriptome of eukaryotic cells and is related to biological activities, such as immunity, inflammation, and carcinogenesis. Previous studies have confirmed that lncRNA could be related to regulation of cell proliferation, differentiation, apoptosis, and invasion in numerous tumors [4, 5]. In addition, lncRNA can interact with microRNA (miRNA) to regulate tumorigenesis and progression. miRNA is a noncoding RNA molecule composed of 20 to 25 nucleotides, which is related to the regulation of cell growth, apoptosis, and migration through binding to target genes. For instance, lnc-SNHG16 was reported to downregulate miR-128 and promote the progression of cervical cancer via inducing the expression of GSPT1 and WNT3A [4]. LINC-PINT suppressed the progression of lung cancer through binding to miR-543 to induce PTEN [6].

Recently, the significance of lncRNA for the diagnosis and treatment of ovarian cancer has attracted much attention [7]. LINC-DUBR is a newly discovered lncRNA, of which the expression reduced in lung adenocarcinoma and inhibited malignant progression [8]. LINC-DUBR impeded the progression of lung adenocarcinoma through binding to ZBTB11 [8]. Nevertheless, whether LINC-DUBR regulates ovarian cancer and its mechanisms have never been reported previously.

We tried to explore the regulation of LINC-DUBR on miR-107 and investigated its effects on the ovarian cancer cells in the present study, aiming to elucidate the biological function of LINC-DUBR in ovarian cancer.

## 2. Materials and Method

### 2.1. Patients and Tissue Specimens

Forty patients with ovarian cancer from February 2017 to January 2019 were collected, all of whom were pathologically confirmed as ovarian cancer, aged 48 to 67 (58.3 ± 5.9) years. All patients received surgical treatment. Ovarian cancer tissues and paracancerous tissues were removed during operation and contained in liquid nitrogen. After the operation, sample tissues were transferred to −80°C refrigerator for storage. All patients who participated in the experiment signed informed consent.

### 2.2. Cell Culture

Normal ovarian epithelial cells HOSE and ovarian cancer cells SKOV3, A2780, and OVCAR3 were purchased from Pricells Co., Ltd, China. SKOV3 was cultured in McCoy's 5A Media (Corning, USA) containing 10% FBS, while HOSE was maintained in DMEM (Thermo Fisher, USA) with 2% fetal bovine serum. All cell lines were maintained in a humidified incubator with 1% penicillin/streptomycin, in a suitable environment with 37°C and 5% CO_2_.

### 2.3. Cell Transfection

miR-107 mimic and inhibitor (GenePharma, China) were adopted for overexpression or knockdown of miR-107. Second mitochondria-derived activator of caspase (SMAC) or LINC-DUBR coding sequence was cloned into pcDNA3.1 (GenePharma, China) for overexpressing SMAC or LINC-DUBR. LINC-DUBR, miR-107 mimic, miR-107 inhibitor, or SMAC were cotransfected into SKOV3 cells by Lipofectamine 2000 reagent (Thermo Fisher Scientific, USA).

### 2.4. RNA Isolation and Quantitative Real-Time PCR Analysis

TRIzol (Tsingke, China) was applied to extract total RNA. After RNA concentration determination, reverse transcription was conducted to obtain cDNA using PrimeScript RT-polymerase (Takara, Japan). The levels of the mRNAs of interest were determined by SYBR Green Premix (Takara, Japan). The primers sequences were synthesized by TsingKe (Shanghai, China).

### 2.5. Western Blot

Total protein was abstracted using Protein Extraction kit (Beyotime Biotechnology, China), and the concentration of protein was analyzed through the BCA assay kit (Thermo Fisher, USA). Proteins were separated using 10% SDS-PAGE gel electrophoresis. Proteins were transferred to the PVDF membrane (Millipore, USA) which was blocked by a mixed solution consisting of 5% milk and PBST for 2 h at 25°C. After that, first antibodies with appropriate dilutions were used to incubate these membranes overnight at 37°C. The membrane was washed through TBST and incubated using secondary antibodies. The protein bands were imaged by the ECL immunoblotting kit (TsingKe, China). The ImageJ-Pro Plus software was applied to measure each of protein bands and then was standardized according to its corresponding *β*-actin band.

### 2.6. CCK-8 Assay

The proliferative capacity was measured using the CCK-8 assay (Dojindo, Japan). A total of 1500 cells per well were added into 96-well plates. These cells were incubated until 24, 48, and 72 hours, and then the absorbance at 450 nm was determined.

### 2.7. Transwell Assay

The transwell assay was conducted to measure cell invasion. 24-well plates with 8 mm polycarbonate filters and chambers (Corning Inc., USA) were used to measure cell invasion. According to the product manual, the filter membrane was covered by Matrigel (BD Biosciences, USA). A total of 5 × 10^5^ cells per well were added into the upper chamber and the lower chamber was added with 600 *μ*L medium. After 24 hours, the cells invading the lower surface through the membrane were fixed using 4% paraformaldehyde, stained, and counted.

### 2.8. Luciferase Reporter Assay

We conducted the luciferase reporter assay to explore the relationship between LINC-DUBR and miR-107. To construct wild-type luciferase reporter vectors named miR-107-WT and the mutant reporter named miR-107-MUT, we inserted the wild-type (WT) or mutant (MUT) miR-107 binding site in 3′UTR into the pGL3 vector (Promega, USA). SKOV3 cells were cotransfected with miR-107-WT or miR-107-MUT and LINC-DUBR by Lipofectamine. Similarly, in order to explore the relationship between miR-107 and SMAC, SKOV3 cells were transfected with miR-107 mimic or negative control, together with SMAC luciferase reporters (wild-type or mutant). Then, the dual-luciferase reporter assay system was used to detected luciferase activity after transfection for 48 h.

### 2.9. Statistical Analysis

The SPSS 20.0 software was applied to analysis all date. *T*-test and one-way ANOVA were applied to figure out the difference between groups. *P* < 0.05 can be considered as that the difference between groups is significant.

## 3. Results

### 3.1. The Expression of LINC-DUBR Decreases in Ovarian Cancer Tissues and Cells

The expression of LINC-DUBR in OC tissue and cell was measured firstly. The results of RT-qPCR showed that LINC-DUBR was lower expressed in OC by comparison with adjacent tissues (Figure 1(a)). LINC-DUBR was observably lower expressed in OC cells (SKOV3, A2780, and OVCAR3) by comparison with HOSE (Figure 1(b)). We chose SKOV3 for follow-up experiment.

### 3.2. Overexpression of LINC-DUBR Impedes Cell Proliferation and Invasion of OC Cells

In order to explore function of LINC-DUBR in ovarian cancer, LINC-DUBR was overexpressed in SKOV3 (Figure 2(a)). Overexpression of LINC-DUBR inhibited the cell proliferation in OC cells SKOV3 (Figures 2(b)). Transwell assay was performed to measure invasive ability of OC cell, and we found overexpressing LINC-DUBR inhibited the invasive ability in OC cells SKOV3 (Figures 2(c) and 2(d)).

### 3.3. LINC-DUBR Directly Regulates the Expression of miR-107

Moreover, TargetScan forecasted that there were binding site between LINC-DUBR and miR-107 (Figure 3(a)). In order to further prove that LINC-DUBR directly regulates miR-107, we carried out luciferase reporter assay, and the results showed LINC-DUBR significantly decreased the luciferase activities of miR-107-WT, but the luciferase activities of miR-107-MUT remained unchanged (Figures 3(b)). Consistently, the expression of miR-107 obviously reduced in LINC-DUBR group and significantly increased in siLINC-DUBR group in ovarian cancer cells SKOV3 (Figures 3(c)).

### 3.4. LINC-DUBR Reverses the Promoting Effect of mir-107 Overexpression on the Proliferation and Invasion of Ovarian Cancer Cells

In order to further prove that LINC-DUBR inhibits progression of OC via regulating miR-107, we measured the miR-107 expression, cell proliferation and invasion after cotransfection of miR-107 mimic and LINC-DUBR into SKOV3. miR-107 mimic observably raised miR-107 expression, but LINC-DUBR inhibited the promoting effect of miR-107 mimic (Figure 3(a)). miR-107 mimic significantly increased cell proliferation (Figure 4(b)) and invasiveness (Figures 4(c) and 4(d)) of SKOV3, while LINC-DUBR eliminated this effect.

### 3.5. miR-107 Directly Downregulated SMAC Expression

TargetScan predicted that SMAC might be the target gene of miR-107 (Figure 5(a)). In order to further prove that miR-107 directly regulates SMAC, we carried out the luciferase reporter assay and results showed miR-107 significantly decreased the luciferase activities of SMAC-WT, but the luciferase activities of SMAC-MUT remained unchanged (Figure 5(b)). Consistently, the expression of SMAC obviously reduced in the miR-107 mimic group and significantly increased in the miR-107 inhibitor group (Figures 5(c) and 5(d)). miR-107 mimic significantly increased cell proliferation (Figure 5(e)) and invasiveness (Figures 5(f) and 5(g)) of SKOV3, while overexpressed SMAC eliminated this effect. In addition, miR-107 overexpression decreased expression of caspase-3 and raised expression of XIAP and overexpressed SMAC eliminated this effect (Figures 5(c), 5(d)).

## 4. Discussion

The pathogenesis of OC is not fully clear, and the significance of epigenetic regulation in OC has been getting more and more attention. lncRNA is a kind of epigenetic regulatory molecule that regulates not only chemical modifications of histones and DNA but also genes in the epigenetic pathway, which fundamentally affect genomic expression.

As a hotspot in the tumor field in recent years, lncRNAs are abnormally expressed in various tumor tissues and is involved in tumorigenic development. For example, LINC00284 targeted MEST to suppress cell proliferation and migration of bladder cancer [9]. LINC-PINT targeted miR-374a-5p to suppress cell proliferation and migration of OC [10]. LINC01006 suppressed the proliferation and invasion of hepatocellular carcinoma cells via regulating miR-433-3p [11]. LINC-DUBR is a newly reported lncRNA and is abnormally expressed in multiple malignancies and suppresses tumorigenesis through multiple pathways [8]. LINC-DUBR was abnormally downregulated and suppressed the malignant progression of lung adenocarcinoma cancer [8]. The present research obtained a similar result which indicated the expression of LINC-DUBR in OC was lower in contrast to adjacent tissues. The relative expression of LINC-DUBR was significantly lower in OC cell lines by comparison with normal cells (HOSE). The proliferative activity and invasiveness of SKOV3 cells were significantly reduced after transfection, suggesting that LINC-DUBR may be associated with the onset and progression of OC.

The mechanism of LINC-DUBR on the progress of tumor has not been fully clarified. The regulatory mechanism of lncRNA on miRNA may be an important way to play its role. Some studies have found that lncRNA targeted miRNAs to regulate the proliferation, invasion, migration and epithelial-mesenchymal transition of tumor cells [12–15]. The prediction results of the TargetScan software showed that miR-107 may be the target gene of LINC-DUBR. We proved that LINC-DUBR directly regulated miR-107 using the luciferase reporter assay. The expression of miR-107 obviously reduced in the LINC-DUBR group and significantly increased in the siLINC-DUBR group in OC cells. miR-107 mimic observably raised cell proliferation and invasiveness of SKOV3, while LINC-DUBR eliminated this effect. These results suggested LINC-DUBR could inhibit the proliferation and invasion of OC cells through targeting miR-107.

In addition, to make clear the mechanism of LINC-DUBR in OC, we proved miR-107 directly regulated SMAC via the luciferase reporter assay. miR-107 significantly reduced the luciferase activities of SMAC-WT, while the luciferase activities of SMAC-MUT remained unchanged. Consistently, the expression of SMAC obviously reduced in the miR-107 mimic group and significantly increased in miR-107 inhibitor group. Furthermore, miR-107 mimic significantly increased cell proliferation and invasiveness of SKOV3, while overexpressed SMAC eliminated this effect. These results suggested that LINC-DUBR may inhibit the proliferation and invasiveness of OC cells via the miR-107/SMAC axis. It has been found that LINC-DUBR could upregulate TMEFF2 expression to inhibit the proliferation of gastric cancer cells by targeting miR-641 [16]. Furthermore, we found miR-107 could regulate the XIAP/caspase-3 signaling pathway in ovarian cancer by targeting SMAC. Caspase-3 is the most important terminal shear enzyme in the process of apoptosis, and it is also an important part of cytotoxic lymphocyte cell killing mechanism. XIAP directly regulates caspase-3/9 to exert its antiapoptotic function [17, 18].

In conclusion, LINC-DUBR suppressed the malignant progression of ovarian cancer by downregulating miR-107 to induce SMAC expression and involving in the XIAP/caspase-3 signaling pathway. LINC-DUBR may become a therapeutic target for ovarian cancer.

## Figures and Tables

**Figure 1:** LINC-DUBR expression in ovarian cancer tissues and cells. (a) Low expression of LINC-DUBR in ovarian cancer tissue (*n* = 40). (b) Low expression of LINC-DUBR in ovarian cancer cells. ^*∗*^*P* < 0.05.

**Figure 2:** Overexpressing LINC-DUBR suppressed progression of ovarian cancer cells. (a) High expression of LINC-DUBR in SKOV3. (b) Suppressing effect of LINC-DUBR on cells proliferation in SKOV3. (c, d) Suppressing effect of LINC-DUBR on cell invision in SKOV3. ^*∗*^*P* < 0.05.

**Figure 3:** LINC-DUBR directly regulates the expression of miR-107. (a) Predicted binding sites. (b) Inhibiting effect of LINC-DUBR on luciferase activity of miR-107-WT in SKOV3 cells. (c) LINC-DUBR regulated the expression of miR-107. ^*∗*^*P* < 0.05.

**Figure 4:** The effect of miR-107 on ovarian cancer progression regulated via LINC-DUBR. (a) The expression of miR-107. (b) LINC-DUBR attenuated promoting the impact of miR-107 mimic on cell proliferation of SKOV3. (c, d). LINC-DUBR attenuated promoting the impact of miR-107 mimic on cell invasiveness of SKOV3. ^*∗*^*P* < 0.05.

**Figure 5:** The effect of SMAC on ovarian cancer progression. (a) Predicted binding sites. (b) Inhibiting effect of miR-107 on luciferase activity of SMAC-WT. (c, d) miR-107 regulated the expression of SMAC, XIAP, and caspase-3. (e) SMAC suppressed the promoting impact of miR-107 on ovarian cancer (OC) cell proliferation. (f, g) SMAC suppressed the promoting impact of miR-107 on OC cell invasiveness. ^*∗*^*P* < 0.05.

## Data Availability

The data to support the findings of this study are available on reasonable request from the corresponding author.
